The article "Biomechanical Analysis of Arm Manipulation in Tai Chi" was published in 2022. Journal: Comput Intell Neurosci.

# Biomechanical Analysis of Arm Manipulation in Tai Chi

**DOI:** 10.1155/2022/2586716

**Published:** 2022-06-17

**Authors:** Xiaoyan Dong, Xiaofan Hu, Biqing Chen

**Affiliations:** ^1^NingboTech University, Zhejiang, Ningbo 315100, China; ^2^Jinhua Polytechnic, Zhejiang, Jinghua 321000, China

## Abstract

In order to explore the kinematics and muscle force characteristics of competitive Taijiquan arm manipulation, and solve the problems of arm trajectory and control in the process of manipulation, this study puts forward the sports biomechanical analysis of arm manipulation in competitive Taijiquan. The technical characteristics and muscle force characteristics of 15 athletes from the competitive Taijiquan team of Xi'an Institute of physical education were studied. Use Excel 2007 and SPSS17.0 to statistically analyze and process the original data. According to the actual needs, the data indicators are summarized. The combined movements of competitive Taijiquan arm manipulation are captured through high-speed photography, and the kinematic data are statistically analyzed, mainly from the two aspects of action amplitude change and action braking. The results show the action track length, relative track length, and action track length of each plane of the two combined hands. The order of the two combined action tracks is: combination 1 > combination 2, in which the action track in the sagittal plane is the longest in combination 1, and it can also be considered that the motion amplitude in the sagittal plane is the largest in combination 1. The average acceleration of group A in the first beat is 0.51 m/s^2^ smaller than that of group B, and the value is 0.22 m/s^2^ smaller. Therefore, the deceleration of group A is larger than that of group B, and the braking capacity of group A is slightly stronger than that of group B. In the second beat, the average acceleration of group B is 1.5722 m/s^2^ larger than that of group A, and the value is 0.210 m/s^2^ larger. The average acceleration of group A in the third, fourth, fifth, and sixth beats is 0.9, 3.728, 0.57, and 0.837 m/s^2^ smaller than that of group B, and the values are 0.466, 0.174, 0.250, and 0.003 m/s^2^ smaller, indicating that the braking capacity of group A in the third, fourth, fifth, sixth, and eighth beats is slightly stronger than that of group B. In the braking of each beat in combination 1 and combination 2 of group AB, the braking ability of arm manipulation of group A is stronger than that of group B. In competitive Taijiquan, the movement techniques of manipulation include: bouncing technology, braking technology, and control technology. For arm manipulation, athletes should have the ability of “braking” technology. In the correlation analysis of movement track length, RMS and I EMG, the score of athletes in group A is high, and there is no correlation between movement track length and RMS. There is a significant correlation between RMS and movement track length in group B, and the correlation degree is moderate. This shows that when the movement of group B athletes is completed, the muscles are in a state of tension, the movement skills are not mastered well, and the energy saving is not achieved. During training, we should pay more attention to the proprioception of muscles and form a correct way of muscle exertion.

The article "Biomechanical Analysis of Arm Manipulation in Tai Chi" was published in 2022. Journal: Comput Intell Neurosci.

## 1. Introduction

After years of experience in the field, the success rate of competitive Taijiquan difficult movements gradually tends to be stable. In the application of difficult movement training methods, professional teams in various provinces and cities are different, but they are developing towards scientific and systematic training. Because the difficult movement of competitive Taijiquan requires one foot landing support, and the connection difficulty coefficient is very large, so that when competitive Taijiquan competition is carried out in the competitive field, there will still be mistakes and points deducted in the difficult movement. Through the investigation on the selection and completion of difficult movements of competitive Taijiquan, this study explores the training methods of difficult movements, so as to contribute to the scientific and sustainable development of competitive Taijiquan in China [1]. From the situation of Chinese competitive Taijiquan competition, the problems of athletes in difficult movements mainly include jumping, shaking, foot rolling, incoherent connection between front and back movements, and so on [2]. Therefore, we should understand the basic characteristics of difficult movements and fully realize the significance of the success of difficult movements for athletes to achieve excellent results. On this basis, the training system of difficult movements of competitive Taijiquan is designed, which has high research value and practical significance for enriching the training methods of difficult movements of competitive Taijiquan. This study summarizes the influencing factors involved in the difficult movement training of competitive Taijiquan, scientifically summarizes and systematically summarizes the methods and steps of difficult movement training of competitive Taijiquan according to the results of questionnaire and interview survey, hoping to provide theoretical basis for improving the overall level of difficult movement completion, find and make up for the shortcomings of difficult movement training methods, and provide theoretical reference for the training practice of competitive Taijiquan [3, 4]. Dynamic analysis is not carried out independently, and it often needs kinematic means to assist it. Synchronous measurement of kinematics and dynamics will better and more scientifically collect and analyze experimental data. Generally, the force value on the body ground or the peak value of flexion and extension muscle group when overcoming resistance can be measured by means of force measuring platform, isokinetic muscle strength tester, and plantar pressure. It is generally used to study the force value at a certain time of a sports event and the explosive power of athletes.  Figure 1 shows the biomechanical factors affecting the economy of running [5].

The article "Biomechanical Analysis of Arm Manipulation in Tai Chi" was published in 2022. Journal: Comput Intell Neurosci.

## 2. Literature Review

Ding et al. used Ariel kinematics video fast feedback analysis system to analyze the three-dimensional kinematics of the rotating shot put technology of two excellent male shot putters in China. The whole action process was divided into six space-time points, and each space-time point was quantitatively analyzed [6]. Acosta and others used the three-dimensional image analysis method to analyze the kinematic characteristics of Chinese professional football players throwing long-distance out of bounds, and came to the conclusion that they want to throw long-distance and high-quality out of bounds. Athletes need to mobilize their body muscles as much as possible for orderly swing from bottom to top, and can release the ball within a reasonable and effective angle range [7]. Lee and others used six optical cameras to obtain the lower limb technical action images of 10 men's volleyball players during the take-off period of front and rear buckle. Through the analysis and research on the kinematic characteristics of the obtained data, it is concluded that the rear spike has shorter take-off time and larger parallel distance than the front buckle. The technical requirements of the front and rear breasting are different in the take-off stage [8]. Peng and others used the biomechanical principle to study and analyze the volleyball spiking action, and concluded that the force order of spiking action [9]. Rodrigues and others believe that testing and analyzing the indexes of kinematics, dynamics, and biology is the main research method and means of sports biomechanics, and the kinematics research method is one of its main research methods [10]. Kim and others have summed up the mechanical principles and requirements of the Taijiquan push hand technical action of “its root is in the foot, hair is in the leg, dominates the waist and shape is in the finger” with mechanical common sense and empirical perception [11]. Sun and others define Taijiquan pushing hand as a competitive skill project that follows certain rules and uses techniques such as hugging, stroking, squeezing, pressing, picking, eight, elbow, and leaning. Both sides stick together, judge each other's strength through the feeling of muscles, and then push each other out with strength to determine the outcome [12]. Anderson and others interpreted Taiji pushing hand as: two people are opponents of each other. According to the principle of “sacrificing themselves to others, calling for smooth delivery, sticking to each other, and not losing the top”, they use the methods of shed, stroking, squeezing, pressing, picking, eight, elbow, leaning, advancing, retreating, looking, looking, and fixing to find out each other's strength and intention through the feeling of their skin, and achieve the form of sports to win each other in an effective way when they have the opportunity and power [13]. Wampler and others described in detail the technical movements of Taijiquan hand pushing, and summarized that the four techniques of holding, stroking, squeezing, and pressing are the main technical movements of Taijiquan hand pushing, which also explains the importance of shed, stroking, squeezing, and pressing in the process of Taijiquan hand pushing [14]. Ahmed and others proposed that Taijiquan push hand is based on the principle of “stick with touch, do not lose, do not top, do not be too short, bend and stretch with bending”, using eight techniques and strength of “shed, stroke, squeeze, press, pick, clear, elbow, and lean”, to practice the sensitivity of skin touch and inner body feeling of limbs, and find out the changes of each other's strength, such as direction, size, rigidity, reality, length, speed, and so on [15].

The article "Biomechanical Analysis of Arm Manipulation in Tai Chi" was published in 2022. Journal: Comput Intell Neurosci.

Based on the current research, this study puts forward the sports biomechanical analysis of arm manipulation in competitive Taijiquan. Using the synchronous measurement method of three-dimensional high-speed camera (casio-fh25) and *s* EMG (megawin6000), this study studies the hand movements of 15 teams in a sports college, evaluates the quality of 15 athletes, and carries out two groups of combined movements. The scores were divided into AB group and statistically analyzed by Excel 2007 and spss170. The results show that in the braking of each beat in combination 1 and combination 2 of group AB, the braking ability of arm manipulation of group A is stronger than that of group B. In competitive Taijiquan, the movement techniques of manipulation include: bouncing technology, braking technology and control technology. For arm manipulation, athletes should have the ability of “braking” technology. In the correlation analysis of movement track length, RMS and *i* EMG, the score of athletes in group A is high, and there is no correlation between movement track length and RMS. There is a significant correlation between RMS and movement track length in group B, and the correlation degree is moderate.

## 3. Method

### 3.1. Research Object

This study takes the technical characteristics and muscle force characteristics of 15 athletes from the competitive Taijiquan team of Xi'an Institute of Physical Education to complete the arm manipulation of competitive Taijiquan.

### 3.2. Research Methods

#### 3.2.1. Subjects

About 15 athletes from the competitive Taijiquan team of a sports college were divided into 4 athletes with grade and 11 athletes without grade, including 10 males and 5 females. And the special years of the subjects were more than 3 years. The height of all subjects was 1.77 ± 0.09 m, the weight was 62.59 ± 8.85 kg, the age was 20.94 ± 1.44 years old, there was no medical history, and the test was in good condition without muscle fatigue. Finally, the athletes are grouped according to the scoring results of the athletes' arm manipulation.

#### 3.2.2. Test Action

The exercise of competitive Taijiquan is complex and changeable, with certain innovation. In the competitive Taijiquan competition, they all appear in the form of combination, so the actions tested in this study are reflected in the form of combination. The arm manipulation of competitive Taijiquan can be divided into: take the shoulder joint as the axis, lift the arm in a certain direction and stop at a certain position, and the range of motion is no more than 180° [16, 17]. Flexion and extension: the upper arm is fixed and the elbow joint is the axis. The elbow joint is extended from straight to curved or from curved to straight. Winding/looping: arc movement of both arms or one arm with the shoulder as the axis or the forearm with the elbow joint as the axis. In the daily training of competitive Taijiquan, the basic arm manipulation movement combination will be practiced, and combined with the basic arm manipulation movement of competitive Taijiquan, so these basic movements are divided into two combination movements. Since the rhythm of the single action structure of winding/looping is not easy to control, the combined action test is not carried out for the action structure of winding. The main actions of combination 1 are: front lift, up lift, side lift, and down lift. The action of combination 2 is also a lift, including side up lift and side down lift. Among them, chest crossing is only a connecting action [18]. In the test, under the unified beat, the beat is 120 beats/minute, and the athletes complete two movements with heel lifting, and take the best group of movements for analysis.

The article "Biomechanical Analysis of Arm Manipulation in Tai Chi" was published in 2022. Journal: Comput Intell Neurosci.

#### 3.2.3. Experimental Equipment

Equipment required for kinematics: 2 CASIO-FH25 high-speed cameras in Japan; Stereo calibration frame; lampstand; Tape measure; 1 synchronous lamp; American APAs image analysis system.

Equipment required by sEMG: Finland megawin6000 surface electromyography wireless remote tester, sampling frequency of 1000 Hz, 17 packs of electromyography, 1 bottle of 75% medical alcohol, 1 shaving knife, and 1 pack of medical tampon.

Equipment required for sEMG standardized test: use Lifefitness and purelength fitness equipment, including pastor chair biceps trainer; Gantry comprehensive trainer; Dumbbells; Sitting high tension back muscle trainer [19].

#### 3.2.4. Experimental Content

Test of high-speed camera: in this test, two high-speed cameras are used for synchronous shooting, and the shooting frequency is 30 Hz to analyze the kinematics of the action image.

Test of actual action sEMG. sEMG test muscles include biceps brachii, triceps brachii, middle bundle of deltoid and latissimus dorsi on the left and right sides, with a total of 8 muscles.

sEMG standardized test.

The maximum random isometric contraction (MIVC) strength test was performed on the tested muscles, and the test results were taken as the standardized value (100%).

#### 3.2.5. Indexes Selected in the Experiment

Kinematic indexes and *s* EMG indexes are selected in this study.

Kinematic index:

Original coordinates: in this study, the original coordinates of each athlete's hand on the *X*, *y* and *Z* axes are selected to calculate the athlete's action track length [20].

Linear speed, this study selects the linear speed from the upper arm to the forearm, and obtains the arm braking effect of each athlete through the change of linear speed.

sEMG indicators:

RMS index, RMS is selected in this study to explore the rhythmicity of motor unit recruitment and excitation of each muscle. The calculation formula of RMS is as follows:

(1) $$\begin{array}{c} RMS=\sqrt{\frac{1}{N}}\sum_{i=1}^{N}X_{i}. \end{array}$$

I EMG index, this study selects iEMG to explore the participation of muscle fibers. The calculation formula is

(2) $$\begin{array}{c} iEMG=\int_{N2}^{N1}X\left(t\right)\text{d}t, \end{array}$$

*N*2 is the starting point of integration; *N*1 is the end point of integration; X(t) is the function value of EMG curve; DT is the sampling interval, in millivolts per second.

#### 3.2.6. Mathematical Statistics

Use Excel 2007 and SPSS17.0 to statistically analyze and process the original data. Summarize various data indicators according to the actual needs. Excel 2007 makes statistics and summary of the data, and uses independent sample *t*-test and correlation analysis to analyze the correlation and difference of the data. If *P* < 0.05, there is significant difference between the mean values of the two samples; if *P* < 0.01, there is very significant difference between the mean values of the two samples [21, 22].

The article "Biomechanical Analysis of Arm Manipulation in Tai Chi" was published in 2022. Journal: Comput Intell Neurosci.

### 3.3. Experimental Process

Two high-speed cameras (casio-fh25, Japan) were used to shoot in the gymnasium of Xi'an Institute of Physical Education by using the method of three-dimensional fixed camera photography. The two cameras and the subjects were in an isosceles right triangle [23]. The shooting distance is 7 m, the machine height is 1.0 m, the focal length is 49 mm, and the shooting frequency is 30 Hz. Use the Finnish MegaWin6000 surface electromyography wireless telemetry system to test it synchronously, and carry out standardized test for each muscle tested.

#### 3.3.1. Test the Main Muscles of the Movement

Analyze the participating muscles of the test action from human anatomy, and analyze the actions of the two combinations, respectively. The results are as follows.

The participating muscles of each action in combination 1: Front lift, up lift, and side lift: biceps brachii, triceps brachii, deltoid, latissimus dorsi, extensor digitorum, extensor ulnaris lateralis, and pectoralis major. Downward lift: biceps brachii, triceps brachii, deltoid, latissimus dorsi, extensor digitorum, and extensor ulnaris lateralis [24].

Participating muscles of each action in combination 2: Chest cross, side down lift: biceps brachii, triceps brachii, deltoid, latissimus dorsi, extensor digitorum, and extensor ulnaris lateralis. Side lift: biceps brachii, triceps brachii, deltoid, latissimus dorsi, extensor digitorum, extensor ulnaris lateralis, and pectoralis major.

#### 3.3.2. Basis of Muscle Selection

The muscles selected in this study are selected according to the structure of human anatomy, muscle function, and the characteristics of surface electromyography wireless remote test system. The biceps brachii spans the shoulder joint, elbow joint, and proximal radioulnar joint, so it has an effect on these three joints. The biceps brachii is divided into long head and short head. The main function is to bend the elbow joint and turn the forearm back [25]. Triceps brachii is located behind the humerus. Its main function is to extend the elbow joint and help the shoulder joint extend back and adduct. The middle bundle of deltoid muscle is located at the shoulder joint, and its main functions are shoulder abduction, flexion and pronation, extension and pronation. Latissimus dorsi is located at the back of the waist and the posterolateral sternum. Its main functions are shoulder joint extension, adduction, and internal rotation.

The article "Biomechanical Analysis of Arm Manipulation in Tai Chi" was published in 2022. Journal: Comput Intell Neurosci.

## 4. Results and Analysis

### 4.1. Kinematic Characteristics of Arm Manipulation

Through high-speed photography, the combined movement of competitive Taijiquan arm manipulation is captured, analyzed by the American APAs image system, and the kinematic data are statistically analyzed, mainly from the two aspects of action amplitude change and action braking. The results are as follows.

#### 4.1.1. Change of Arm Manipulation Range

In competitive Taijiquan, the range of movement is one of the standards to judge the quality of athletes' movement completion. Action trajectory refers to the spatial characteristics of the action composed of the route that a part of the body passes from the starting position to the end. In kinematics, the length of action trajectory can be used to reflect the size of action amplitude. In arm manipulation, there are “route” requirements for combined action. The “route” of an action is the trajectory from one action to another. If the combination of manipulation action is straight arm, it is required to take the farthest “route”. If the arm action is from bending arm to straight arm, it is required to take the shortest “route”. In this study, because the athletes have a long sports life and the action routes of combined actions meet the above requirements, the action amplitude of combined actions of groups A and B is analyzed by the length of action track in biomechanics. The calculation of the length of the action track is based on the original coordinates of the athlete's completion of the action. The length from the second coordinate point to the first coordinate point is obtained, then it is superimposed, and finally the sum is obtained to obtain the track length of the complete action. Available formula is as follows:

(3) $$\begin{array}{c} L=\sum \sqrt{{\left(X_{n+1}+X_{n}\right)}^{2}+{\left(Y_{n+1}-Y_{n}\right)}^{2}+{\left(Z_{n+1}-Z_{n}\right)}^{2}},n=1,2,3,\ldots , \end{array}$$

where *L* is the length of action track.

The hand is the limb end of the arm, and the movement track of the hand can be regarded as the movement track of each combined action. The track length of an athlete can also represent the range of motion of the athlete. In this study, the movement trajectory of the hand is selected, the trajectory length of the left and right hands is calculated, respectively, and then the average value is taken to reflect the trajectory length of the athlete's movement in the combination. Due to the difference of gender and height, the relative track length is obtained by the ratio of action track length to height. In order to more intuitively understand the movement trajectory changes of each combined action, select the movement trajectory of Jiang's left and right hands in group A and Niu's left and right hands in group B.

The article "Biomechanical Analysis of Arm Manipulation in Tai Chi" was published in 2022. Journal: Comput Intell Neurosci.

It can be seen from Table 1 that there is no significant difference between the two groups from the results of *t*-test. According to the action structure, the combined actions include flexion, abduction, adduction, and so on. In terms of numerical value, group A was longer than group B in terms of track length in horizontal plane, sagittal plane, frontal plane, and relative track length. In terms of relative track length, group A is 19.2 cm longer than group B on the sagittal plane, 7.5 cm longer than group B on the frontal plane, and 13.5 cm longer than group B on the horizontal plane. The longest length of group A is in the sagittal plane, and the longest length of group B is in the frontal plane. In combination I, the action amplitude of group A is greater than that of group B. It can be considered that the combined action has a long trajectory in the frontal and sagittal planes.

This is due to the action structure. The first four beats and the last four beats of the combined action of combination I are symmetrical actions, in which the front lift (the first beat and the seventh beat) and the up lift (the second beat and the sixth beat) mainly move in the frontal plane and horizontal plane, and the side lift (the third beat and the fifth beat) and the down lift (the fourth beat and the eighth beat) mainly move in the sagittal plane and horizontal plane. Combined with the relative track length, the action amplitude of group A in front lift and up lift is greater than that in side lift and down lift. The range of side lift and down lift in group B was greater than that in front lift and side lift.

The action trajectories of the two groups of hands are different on each plane, so the statistical analysis of the trajectories of XY (horizontal plane), XZ (frontal plane), and YZ (sagittal plane) on each plane is shown in Table 2.

It can be seen from Table 2 that there is no significant difference between the two groups from the results of *t*-test. According to the action structure, the actions of combination 2 include flexion, external rotation, adduction, and so on. In terms of numerical value, group A was longer than group B in terms of track length in horizontal plane, sagittal plane, frontal plane, and relative track length. From the perspective of relative trajectory, the longest is in the horizontal plane. On the horizontal plane, group A is 34.8 cm longer than group B. Secondly, in the sagittal plane, group A was 11 cm longer than group B. The shortest length was on the frontal plane. Group A was 8.1 cm longer than group B. It can be considered that in combination 2, the trajectory of motion on the horizontal plane is the longest. This is due to the structure of the action. The combination two has four beats, in which the chest cross two beats (the first beat and the third beat) mainly move in the horizontal plane and sagittal plane. The action structure of side up lift and side down lift is the same, but the end position of the action is different. One is side up (45° inclined up) and the other is side down (45° inclined down). Its moving surface is the same. The two beat actions move on the frontal plane and horizontal plane. Combined with the action structure and research results, it shows that the combined action of combination 2 has the longest trajectory on the horizontal plane, that is, the maximum motion amplitude on the horizontal plane.

The article "Biomechanical Analysis of Arm Manipulation in Tai Chi" was published in 2022. Journal: Comput Intell Neurosci.

Based on the above, the action track length, relative track length, and action track length of each plane of the two combined hands. The order of the two combined action tracks is: combination 1 > combination 2, in which the action track in the sagittal plane is the longest in combination 1, and it can also be considered that the motion amplitude in the sagittal plane is the largest in combination 1. The action track of combination 2 is the longest on the horizontal plane, and it is considered that the movement amplitude of combination 2 is the largest on the horizontal plane. In the action trajectories of these two combinations, the action trajectories of group A are longer than those of group B, and the action range of group A is larger than that of group B in the three combinations, which is consistent with the score results of the referee. Therefore, the length of action trajectories can be used as one of the criteria for judging the arm manipulation of athletes. The reason for the difference between the action trajectories of the two combined actions is that the beat is inconsistent: among them, combination 1 is an eight beat action and combination 2 is a four beat action. Difference of action structure: because each combined action structure has its own characteristics, the motion trajectory of each combination is different. Combined with the height difference between the two groups of athletes, there is no significant difference. The difference between the mean values is only 0.94 cm, and the movement structure is consistent. The reason for the difference in the length of movement track between the two groups of AB is that the movement of group B athletes is not “in place”. In particular, the action of lifting requires a certain angle of arm action. For example, the forward lift requires the arm to be parallel to the ground when the action is in place, and the upward lift requires the arm to be located on the ear side. In training, the coach requires the “arm to clamp the ear”. The action route is not clear: in competitive Taijiquan, the action of lifting requires taking the “farthest route”. For example, in combination 1, the “farthest route” should be taken from the front lift to the upper lift, and the same is true from the upper lift to the side lift. Some of these movements require the most recent route. Flexibility of shoulder: from the results, the movement track length of group B is smaller than that of group A, indicating that the flexibility of group A's shoulder is better than that of group B. When athletes do movements, they shrug and pinch their shoulders, especially when their arms are up. Some athletes are used to shrugging their shoulders. For this phenomenon, athletes should strengthen the practice of proprioception, always remind when doing actions, and slowly correct this wrong habit.

The article "Biomechanical Analysis of Arm Manipulation in Tai Chi" was published in 2022. Journal: Comput Intell Neurosci.

#### 4.1.2. Arm Action Braking Effect

In competitive Taijiquan, whether the arm manipulation action of a single action or the combined arm manipulation action, each beat action needs to have “braking”. In the kinematic index, the change of midline speed can be reflected from the moment of maximum online speed to the end of the action or the moment when the speed drops to zero. The speed change during this period is the “braking” of the arm, which is expressed by Δ*v* and the average acceleration $\bar{a}$, according to the formula

(4) $$\begin{array}{c} \bar{a}=\frac{\Delta v}{\Delta t}. \end{array}$$

Through the index of linear speed, the Δ*v* value and average acceleration of each athlete's left hand and right hand in each beat are calculated, and then the average value is taken. The mean value can be considered as the speed change during the braking of the athlete's arm movement. The results of Δ*v* and average acceleration of each beat between the two groups are shown in Tables 3 and 4.

The arm braking changes and *t*-test results of each beat in combination I are shown in Table 3. It can be seen from Table 3 that in terms of speed change, the minus sign only represents the deceleration process. In terms of value, the change trend of the two groups of speeds is consistent with the acceleration. The average acceleration of group A in the first beat is 0.51 m/s^2^ smaller than that of group B, and the Δ*v* value is 0.22 m/s^2^ smaller. Therefore, the deceleration of group A is larger than that of group B, and the braking capacity of group A is slightly stronger than that of group B. In the second beat, the average acceleration of group B is 1.5722 m/s^2^ greater than that of group A, and the Δ*v* value is 0.210 m/s^2^ greater. The average acceleration of group A in the third, fourth, fifth, and sixth beats is 0.9, 3.728, 0.57, and 0.837 m/s^2^ smaller than that of group B, and the V value is 0.466, 0.174, 0.25,0 and 0.003 m/s^2^ smaller, indicating that the braking capacity of group A in the third, fourth, fifth, sixt,h and eighth beats is slightly stronger than that of group B. The Δ*v* value and average acceleration of group B in the seventh beat are less than those of group A. It can be considered that the braking capacity of group B in the seventh beat is slightly stronger than that of group A. The Δ*v* value and average acceleration of group A in the eighth beat are smaller than those of group B, the deceleration of group B in the eighth beat is larger than that of group A, and the braking capacity of group A is slightly stronger than that of group B. It can be seen from the above that in the eight beat action of combination 1, the braking ability of group A is stronger than that of group B in the six beat action, and the braking ability of group B in the two beat action is stronger than that of group A. It can be considered that in the combination action of combination 1, the braking ability of athletes in group A is stronger than that of group B. The braking action of the second and seventh beats is the change between the front lift and the up lift. The braking action of the second beat is the braking action from the front lift to the upper lift, and the braking action of the seventh beat is the braking action from the upper lift to the front lift. The changes between the two movements of the athletes in group A are not as good as those in group B. The braking capacity of other actions of group B is not as good as that of group A.

The article "Biomechanical Analysis of Arm Manipulation in Tai Chi" was published in 2022. Journal: Comput Intell Neurosci.

In combination 2, the braking changes of the arm at each beat are shown in Table 4. It can be seen from Table 4 that from the numerical point of view, the change trend of the two groups of speeds is consistent with the acceleration. The Δ*v* value and average acceleration of the first, second, and fourth beat actions of group A are less than those of group B. from the perspective of braking effect, the braking ability of the arm manipulation combination actions of group A of the first, second, and fourth beat is stronger than that of group B. The Δ*v* value and average acceleration of group B in the third beat are less than that of group A. From the perspective of braking effect, the braking ability of group B in the third beat is better than that of group A. The braking of the third beat is the action of lifting from the side up to the chest cross. In this beat, the braking of group A is stronger than that of group B. On the whole, in combination 2, the braking ability of arm manipulation in group A is stronger than that in group B, and the arm manipulation braking technology in group A is better than that in group B.

Based on the above data results, from the results of *t*-test, there is no significant difference between AB and ab groups (*P* > 0.05). From the numerical point of view, in the braking of each beat in combination 1 and combination 2 of group AB, the braking ability of arm manipulation of group A is stronger than that of group B. In competitive Taijiquan, the movement techniques of manipulation include: bouncing technology, braking technology and control technology. For arm manipulation, athletes should have the ability of “braking” technology. Through the braking technology, we can see the athlete's control over the action, and through the action control ability, we can evaluate the athlete's ability and level. Generally speaking, athletes with good action braking ability also have a good grasp of action control and understanding. The braking ability of the movement also reflects the athlete's control of muscle tension and relaxation. From the formation process of motor skills, it shows that the inhibition of motor center in cerebral cortex has been established and the formation of motor skills is automatic. The braking ability of group B athletes is weaker than that of group A. the main reasons are: the muscle exertion mode is wrong: the main exerting muscles of group AB athletes may be different, so there are differences in the muscle parts of action exertion. There are differences in muscle tension and relaxation ability: in competitive Taijiquan, athletes need to exert force and brake quickly, and have high requirements for muscle tension and relaxation ability. The ability of muscle tension and relaxation can be called energy saving in physiology. The ability of excellent athletes in this aspect is greater than that of ordinary athletes. There are some wrong movements: because the sports years of the two groups of athletes are more than three years, the movements have been automated. The original wrong action has also become automatic and difficult to correct.

### 4.2. s EMG Analysis

The *s* EMG of this study was carried out simultaneously with high-speed photography to explore the muscle force characteristics of athletes in each combination. The main muscles tested are: left biceps brachii, left triceps brachii, left deltoid middle bundle, left latissimus dorsi, right biceps brachii, right triceps brachii, right deltoid middle bundle, and right latissimus dorsi. RMS and EMG were selected to judge the strength of each muscle activity. Considering the difference of sebum thickness among athletes, it is impossible to make a direct comparative analysis. In the process of the experiment, each muscle is standardized, and then the standardized value of each athlete is obtained, and of each athlete is compared and analyzed.

The article "Biomechanical Analysis of Arm Manipulation in Tai Chi" was published in 2022. Journal: Comput Intell Neurosci.

#### 4.2.1. Combination 1 s EMG Feature

The standardized value of RMS of combination 1 is shown in Figure 2.

As can be seen from Figure 2, the maximum muscles of the two groups are different. Group A is 118.87% of the right latissimus dorsi, group B is 75.78% of the left triceps brachii, and the minimum muscles are the left biceps brachii, group A is 12.87%, and group B is 10.78%. From the above figure, we can see that the standardized values of the muscles and standardized actions on the right are larger than those on the left. In group A, the latissimus dorsi and triceps brachii on both sides and biceps brachii were larger than those in group B, and the RMS standardized values of other muscles in group B were larger than those in group A.

The *i* EMG features of the combination are shown in Figure 3.

It can be seen from Figure 3 that in the combined arm manipulation, the standardized values of latissimus dorsi on both sides of group A are larger than those of other muscles, and the standardized values of triceps brachii on the left and biceps brachii on the right in group B are larger than those of other muscles. The lowest standardized value of the two groups was the left biceps brachii.

Based on the above standardized values of RMS and I EMG, the muscle standardized values of the two groups changed, but the change trend of their standardized size was unchanged. In the exercise of combination 1, the arms on both sides start to act at the same time. It is found that the standardized value of athletes in group AB is greater on the right than on the left. This is because the dominant hand of most athletes is the right hand, which is related to personal sports habits. Combined with the standardized values of RMS and I EMG in Figures 3 and 4, it is found that the recruitment ability and excitation rhythm of motor units of latissimus dorsi muscle in group A are stronger than those of other muscles, and the participation of muscle fibers is also more than that of other muscles. It can be considered that the latissimus dorsi muscle is the main muscle involved in the arm manipulation of group A, and the triceps brachii on the left and biceps brachii on the right in group B have stronger recruitment ability and excitation rhythm of motor units than other muscles, and the participation of muscle fibers is also more than other muscles. It can be considered that the main muscles in group B are the triceps brachii on the left and the biceps brachii on the right. Combined with the scoring results of the referees on the athletes' arm manipulation movement, the athletes in group A are higher than those in group B, which shows that the action completion quality of group A is high, and it can be considered that the action force mode of this group of athletes is more correct than that of group B. Therefore, the main muscles of combined arm manipulation are latissimus dorsi on both sides. The athletes in group B should improve the way of exertion, no longer take the left triceps brachii and the right biceps brachii as the main exerting muscles, but change to latissimus dorsi.

The article "Biomechanical Analysis of Arm Manipulation in Tai Chi" was published in 2022. Journal: Comput Intell Neurosci.

#### 4.2.2. sEMG Characteristics of Combination 2

The standardized value of RMS of combination 2 is shown in Figure 4.

As can be seen from Figure 4, among the standardized values of all muscles in group A, the maximum value is 89.61% of the latissimus dorsi on the right, and the minimum value is 11.32% of the biceps brachii on the left. Among the standardized values of all muscles in group B, the maximum value was 56.31% of the biceps brachii on the right and the minimum value was 17.69% of the latissimus dorsi on the left. The RMS standardized values of bilateral latissimus dorsi, right triceps brachii, and middle bundle of right deltoid in group A were higher than those in group B. In general, the standardized value of the right muscle in group A was greater than that in group B, and the standardized value of the left muscle in group B was greater than that in group A.

The *i* EMG characteristics of combination II are shown in Figure 5.

As shown in Figure 5, in the combined second-hand arm manipulation, the standardized value of latissimus dorsi on both sides of group A is the largest, and the lowest standardized value is the left biceps brachii. In group B, the standardized values of the left triceps brachii and the right biceps brachii were greater than those of other muscles, and the smallest value was the left latissimus dorsi.

Based on the above standardized values of RMS and I EMG, the muscle standardized values of the two groups changed, but the change trend of their standardized size was unchanged. It is found that the muscle force on the right side of the athletes in group AB is greater than that on the left, indicating that the dominant hand of both groups is the right hand. This is because the dominant hand of most athletes is the right hand, which is related to personal sports habits. Combined with the standardized values of RMS and I EMG of latissimus dorsi in Figures 4 and 5, it is found that the recruitment ability and excitation rhythm of motor units of latissimus dorsi in group A are stronger than those of other muscles, and the participation of muscle fibers is also more than that of other muscles. It can be considered that in the arm manipulation of combination 2, the latissimus dorsi muscle is the main muscle involved in group A, and the recruitment ability and excitation rhythm of motor units of right biceps brachii and left triceps brachii in group B are stronger than those of other muscles, and the participation of muscle fibers is also more than that of other muscles. It can be considered that the main muscles in group B are the right biceps brachii and the left triceps brachii. Combined with the score results of the referee on the athletes' arm manipulation movement, it shows that the movement completion quality of group A is high, and it can be considered that the movement force mode of this group of athletes is more correct than that of group B. Therefore, the main muscles for the arm manipulation of combination 2 are the latissimus dorsi muscles on the left and right sides.

The article "Biomechanical Analysis of Arm Manipulation in Tai Chi" was published in 2022. Journal: Comput Intell Neurosci.

According to the characteristics of RMS and *i* EMG in these two combinations, the latissimus dorsi muscle is the main muscle in group A in the three combinations. The main muscles involved in group B in combinations 1 and 2 are the right triceps brachii and the left biceps brachii. In competitive Taijiquan, the basic form requirements for athletes are: lift the heels of both feet, clamp the legs and hips inward, clamp the shoulder blades backward, straighten the spine, sink the shoulders, center the head, open both hands, straighten the arms, put the five fingers together, and force to the fingertips. The control of athletes' basic posture also reflects the control ability of athletes to a certain extent. Combined with the structure and function of muscles and the research results, it can be considered that the basic shape of group A is better than group B, and the control ability of group A is stronger than group B. From the perspective of sports skills, the athletes in group A have a high degree of energy saving, good nerve control over muscles, and less redundant actions. It is suggested that athletes and coaches should mainly focus on the training of latissimus dorsi muscle in the training of arm manipulation, instead of the traditional arm muscle strength training.

In the correlation analysis of motion trajectory length, RMS and *i* EMG, there was no linear correlation in group A and moderate correlation in group B. The correlation between action track length and RMS and *i* EMG in group B was greater than that in group A. Combined with the referee's score results, the athletes in group A have high scores, and there is no correlation between the three indexes of action track length and RMS. There is a significant correlation between RMS and movement track length in group B, and the correlation degree is moderate. This shows that when the movement of group B athletes is completed, the muscles are in a state of tension, the movement skills are not mastered well, and the energy saving is not achieved. During training, we should pay more attention to the proprioception of muscles and form a correct way of muscle exertion.

The article "Biomechanical Analysis of Arm Manipulation in Tai Chi" was published in 2022. Journal: Comput Intell Neurosci.

## 5. Conclusion

This study provides a biomechanical analysis of the movements of Taijiquan hands. In this study, biomechanical research methods and tools were used to analyze the arm manipulation of competitive Taijiquan, and the problems of kinematics and muscle strength characteristics were solved. Pull and control arm movement during adjustment. Using the synchronous measurement method of three-dimensional high-speed camera (casio-fh25) and *s* EMG (megawin6000), this study studies the hand movements of 15 teams in a sports college, evaluates the quality of 15 athletes, and carries out two groups of combined movements. The scores were divided into AB group and statistically analyzed by Excel 2007 and spss170. The kinematic characteristics of arm exercise and the strength characteristics of eight muscles (biceps, triceps, middle deltoid, and major muscle) were studied in the two groups of athletes. The results show that in the competitive Taijiquan movement combining hand and chemistry, the movement of group a athletes is close to the music rhythm, and the movement coordination conforms to the rhythm of group A, which is more than that of group B. The larger the relative trajectory, the greater the motion amplitude and the higher the elongation. The length of track a is longer than that of group B, which is consistent with the scoring results. The “braking” method is very important. Comparing the normal values of RMS and I EMG during ab exercise between the two groups, the right muscle load was greater than the left. When combined with arm exercises, the core muscles use the left and right back muscles. The main muscles in group A are back muscles, and the main muscles in group B are triceps and biceps. In order to further brake the hand action, you can switch the hand action from two times to one blow, and feel the braking process. For athletes who have completed the action automation, special attention should be paid to the “in place” of the action.

The article "Biomechanical Analysis of Arm Manipulation in Tai Chi" was published in 2022. Journal: Comput Intell Neurosci.

## Figures and Tables

**Figure 1:** Biomechanical factors affecting running economy. It is generally used to study the force value at a certain time of a sports event and the explosive power of athletes.

**Figure 2:** RMS standardized values of muscles in group AB. In group A the latissimus dorsi and triceps brachii on both sides and biceps brachii were larger than those in group B and the RMS standardized values of other muscles in group B were larger than those in group A.

**Figure 3:** Standardized values of I EMG of muscles in groups B and AB. The lowest standardized value of the two groups was the left biceps brachii.

**Figure 4:** RMS standardized values of muscles in group AB. Among the standardized values of all muscles in group (B) the maximum value was 56.31% of the biceps brachii on the right and the minimum value was 17.69% of the latissimus dorsi on the left.

**Figure 5:** Standardized values of i EMG of muscles in group AB. In group B the standardized values of the left triceps brachii and the right biceps brachii were greater than those of other muscles, and the smallest value was the left latissimus dorsi.

**Table 1:** Track length of group AB hand.

	*XY*	*XZ*	*YZ*
Group a track length	6.076 ± 0.531	7.467 ± 0.442	7.572 ± 0.456
Group B track length	5.869 ± 0.29	7.382 ± 0.357	7.278 ± 0.344
Difference (A-B)	0.194	0.086	0.275
Group a relative track length	3.545 ± 0.384	4.362 ± 0.330	4.424 ± 0.349
Group B relative track length	3.412 ± 0.175	4.285 ± 0.202	4.24 ± 0.255
Difference (A-B)	0.136	0.076	0.193

**Table 2:** Action track length of group AB hands.

	*XY*	*XZ*	*YZ*
Group A track length	5.182 ± 0.576	4.548 ± 0.288	4.598 ± 0.53
Group B track length	4.617 ± 0.476	4.386 ± 0.387	4.428 ± 0.472
Difference (A-B)	0.568	0.163	0.169
Group A relative track length	3.032 ± 0.400	2.658 ± 0.238	2.689 ± 0.238
Group B relative track length	2.684 ± 0.299	2.548 ± 0.23	2.577 ± 0.318
Difference (A-B)	0.349	0.12	0.082

**Table 3:** Arm action braking of group AB.

Rhythm	1	2	3	4	5	6	7	8
Group A Δ*v*	−3.498 ± 0.704	−2.869 ± 0.737	−3.404 ± 0.843	−3.809 ± 0.775	−3.938 ± 1	−3.12 ± 0.76	−3.16 ± 1.2	−3.51 ± 1.02
Group B Δ*v*	−3.269 ± 0.663	−3.054 ± 0.376	−2.941 ± 0.531	−3.635 ± 0.517	−3.681 ± 10.61	−3.13 ± 0.3	−3.1 ± 0.41	−3.21 ± 0.39
Difference A-B Δ*v*	−0.228	0.186	−0.466	−0.172	−0.258	−0.002	0.06	−0.29
Group A $\bar{a}$	−17.643 ± 12.356	−13.422 ± 7.461	−16.877 ± 9.708	−22.936 ± 9.374	−18.772 ± 11.67	−17.91 ± 10.78	−16.43 ± 11.04	−16.04 ± 12.34
Group B $\bar{a}$	−17.143 ± 5.862	−14.993 ± 3.215	−16.173 ± 5.328	−19.207 ± 11.54	−18.21 ± 5.33	−17.08 ± 4.48	−17.99 ± 6.36	−14.71 ± 3.24
Difference A-B $\bar{a}$	−0.6	1.572	−0.8	−3.726	−0.57	−0.837	1.567	−1.335

The article "Biomechanical Analysis of Arm Manipulation in Tai Chi" was published in 2022. Journal: Comput Intell Neurosci.

**Table 4:** Arm action braking of group AB.

Rhythm	1	2	3	4
Group A Δ*v*	−3.498 ± 0.31	−3.72 ± 2.44	−9.8 ± 0.44	−5.18 ± 1.29
Group B Δ*v*	−4.09 ± 0.99	−3.26 ± 0.49	−8.56 ± 0.43	−4.72 ± 0.8
Difference A-B Δ*v*	−0.7	−0.46	−1.24	−0.45
Group A $\bar{a}$	−14.88 ± 6.12	−23.82 ± 17.47	−13.42 ± 7.46	−19.67 ± 9.38
Group B $\bar{a}$	−13.46 ± 5.32	−18.22 ± 7.94	−14.7 ± 4.44	−19.18 ± 8.58
Difference A-B $\bar{a}$	−1.41	−5.6	−1.27	−4.99

## Data Availability

The data used to support the findings of this study are available from the corresponding author upon request.
